This article has been retracted.

# A Novel Artificial Intelligence System in Formulation Dissolution Prediction

**DOI:** 10.1155/2022/8640115

**Published:** 2022-08-08

**Authors:** Haoyu Wang, Chiew Foong Kwong, Qianyu Liu, Zhixin Liu, Zhiyuan Chen

**Affiliations:** ^1^Department of Electrical and Electronic Engineering, University of Nottingham Ningbo China, Ningbo, China; ^2^International Doctoral Innovation Centre, NingboTech University, Ningbo, China; ^3^Department of Outpatient, Liaoning Thrombus Treatment Center of Integrated Chinese and Western Medicine, Shenyang, China; ^4^Department of Mechanical, Materials and Manufacture, University of Nottingham Ningbo China, Ningbo, China

## Abstract

Artificial neural network (ANN) techniques are widely used to screen the data and predict the experimental result in pharmaceutical studies. In this study, a novel dissolution result prediction and screen system with a backpropagation network and regression methods was modeled. For this purpose, 21 groups of dissolution data were used to train and verify the ANN model. Based on the design of input data, the related data were still available to train the ANN model when the formulation composition was changed. Two regression methods, the effective data regression method (EDRM) and the reference line regression method (RLRM), make this system predict dissolution results with a high accuracy rate but use less database than the orthogonal experiment. Based on the decision tree, a data screen function is also realized in this system. This ANN model provides a novel drug prediction system with a decrease in time and cost and also easily facilitates the design of new formulation.

## 1. Introduction and Background

The computational method is an important alternative to the experimental method. By analyzing and calculating drug sequence data [1], a machine learning algorithm is used to predict drug solubility [2]. Commonly used machine learning algorithms are mainly support-vector machine [3], neural network algorithm [4], random forest [5], and other methods. CCSOL [6] is a SVM-based prediction tool established by Federico et al. in 2012, and it was first proposed to use hydrophobicity, *β* folding, and *α* helix as the main features. Parsnip [7] was a tool published by REDA et al. in 2017. Meanwhile, it was proposed that a high proportion of exposed residues was positively correlated with drug solubility, and tripeptides composed of multiple histidine and tripeptide fragments were negatively correlated with drug solubility. SOLpro [8] extracted 23 groups of features from the first-level sequence for training the two-stage support-vector machine (SVM) architecture. PROSOII [9] is a second-level logical classifier with modified a Cauchy kernel probability density window model used by PAWEL et al. However, most existing studies use the SVM model as the classifier, which has limited processing ability and slow speed for big data. Deep learning is the core field of artificial intelligence technology at present [10]. Compared with “shallow learning” such as SVM, the deep learning model can obtain more nonlinear relations [11]. The convolutional neural network is one of the important frameworks of deep learning. It has been widely applied in image detection [12], face recognition [13], audio retrieval [14] and achieved good results, but it is seldom applied in the research field of drug solubility prediction. Sameerkhurana et al.[15] of MIT constructed the DeepSol prediction model in 2018. One-hot was mainly used to encode drug sequences, and 21 *∗* 1200 feature matrix was obtained. A shallow parallel convolutional neural network model with seven convolution kernels of different sizes was established to predict drug solubility.

The formulation is made to meet the needs of treatment or prevention according to specific dosage form requirements. A formulation is a medicine that can be finally provided to the subject for use. The formulation has different dosage forms, such as tablets, pills, powders, tinctures, patches, injections, aerosols, sprays, ointments, and suppositories. The main dosage research of this project is tablets [16].

This project is the focus on the prediction of formulation dissolution result during the changing of formulation compositions. The recent research work comparison is shown in Table 1.

As shown in the table, the regression method of others' work cannot satisfy the stability of the prediction result due to the prediction times and the regression method. In this project, both methods include the function of screening abnormal prediction results before regressing. In addition, in comparison, this project uses a small amount of input data that achieved accurate prediction. In addition, there are three kinds of formulation composition in this experiment. The related experimental data are still valid, although the formulation composition is changed in the model.

In an experiment process, experimental design is an important optimization. The design and production of experiments require researchers to predict the next step of the planned process in the following experiment and then conduct experiments to reduce the number of experiments and increase the efficiency of the quantity project based on the experiments. However, human prediction requires a large amount of experience, and its results also have partial results prediction, so it is impossible to successfully predict the possibility. Optimization requires 100 or more experiments to complete, so researchers cannot import massive data for analysis [20].

Existing formulation prediction software mainly uses linear regression algorithms for calculation. The algorithm is simple. For the simulation of the dissolution of the preparation, accurate prediction can be achieved when the data difference is not significant. However, when the data significantly change, its accuracy will be significantly reduced. Second, the existing formulation prediction software needs to input a large amount of data to fit the curve before each prediction, perform the curve correction automatically or manually, and then start the prediction. Although the more considerable the amount of data, the higher the accuracy. However, because the linear regression algorithm cannot solve the nonlinear problem of the dissolution of the preparation, there is always a bottleneck in prediction accuracy. When it reaches a certain level, the amount of data will not increase if it is increased. For some applications of AI used in formulation prediction, they always use a large amount of data to train the model. Then, they can receive a prediction result from the model. The problem is that, when the experimental result reaches that amount, the project is nearly complete [21]. The prediction becomes meaningless.

This project uses machine learning methods in artificial intelligence, uses a neural network to solve nonlinear problems, establishes a mathematical model, and uses experimental data to train the model. In this project, all the influencing factors in the experiment are digitized, including prescription ratio, preparation process parameters, equipment parameters, and batch size. Compared with traditional linear prediction methods, this method requires a large amount of known data for training, but the requirements for training data are entirely different. The training data required by this method only need to be the preparation development data related to the prediction. For example, experiment data with the same or similar excipients as the target formulation can also be the input data. In addition, the system can also become an “omnipotent wise man” under the training of high-throughput data. The trained model can predict any related formulation variety under the premise of a small number of experiments.

The feature of this project is that when the input data are insufficient, the results can also be predicted through algorithms. In order to collect more data during the practical applications, a method is designed in this model to achieve when the prescription excipients are fine-tuned. The previous similar data can still be used as input data to train the model. In addition, the problems that may be encountered in future high-throughput data input are also studied. First, there will inevitably be abnormal data due to operator errors and other reasons due to a large amount of data. Therefore, the automatic data input method of this project is optimized. We use artificial intelligence methods to detect input data and provide manual or automatic screening functions.

## 2. Materials and Methods

### 2.1. Materials

The composition for tinidazole is given in Table 2.

### 2.2. Tinidazole Tablet Preparation

The main step of tinidazole tablet preparation can be described in 7 steps:

 
*Step 1*. API treatment: we put the tinidazole powder into a vacuum-drying oven and dry it under reduced pressure for 2 hours at a temperature of 60°C and pressure of 1 kPa. After natural cooling in a low-pressure environment of 1 kPa, the API is taken out, then put into a grinder for pulverization, and sieved.
 
*Step 2*. Preparation of the adhesive: we weigh the prescription amount of HPMC, add part of the boiling water, and then use a glass rod to continuously stir until the HPMC is completely dispersed in the liquid. Then, we use room temperature water to make up the remaining prescription water, continue to stir for 30 minutes, and then stand for 12 hours.
 
*Step 3*. Total mixing: the tinidazole API is mixed with inactive ingredients except for the binder and magnesium stearate, put into the *V*-type mixer, and mixed for 30 minutes.
 
*Step 4.* Granulation: we put the mixed sample into the granulator, turn on the shearing knife, and slowly add the binder.
 
*Step 5.* Drying: after the granulation, the granules are put into the tray. The tray is put into the oven to dry until the moisture content is qualified.
 
*Step 6*. Granules: we put the dried granules into the finishing machine for granulation.
 
*Step 7.* Compressing tablets: we add magnesium stearate to the whole granules, put them in a *V*-type mixer, and mix for 5 minutes. We adjust the tablet press speed, precompression parameters and tablet thickness parameters, and start tablet compression.

### 2.3. Model Test Design

First, a formulation experiment with different prescriptions and prescription quantities is designed to test the model's adaptability. Due to the small amount of training data, the results of each prediction greatly vary, which affects the accuracy of the prediction [22, 23]. Therefore, the regression value is calculated after multiple predictions to process the predicted value. In addition, we designed a gradient experiment that is designed to verify the improvement of prediction accuracy when the amount of input data increases. Due to the limited experimental conditions, 21 sets of prescriptions and dissolution data with three different excipients were used in this test.

Therefore, the test is divided into three parts. The first part is to test the impact of training times on the stability of the result; the second part is to test the impact of the training dataset on the prediction accuracy; and the third part is to make predictions on 21 sets of data to test their experimental adaptability.

### 2.4. Artificial Neural Network (ANN) Design

The critical elements of this project are the prescription ratio, the dissolution time, and the dissolution rate at each time point (percentage of drug dissolution in different time points). To establish connections among time points, the formulation ratio and the dissolution time were set as the input data set and the dissolution rate at each time point was set as the output data.

In Figure 1, the *X*1–*X*8 mean the following: *X*1, time value (minutes) of dissolution test; *X*2, percentage of tinidazole; *X*3, percentage of microcrystalline cellulose PH 101; *X*4, percentage of starch; *X*5, percentage of croscarmellose sodium; *X*6, percentage of hydroxypropyl methylcellulose; *X*7, percentage of magnesium stearate; and *X*8, percentage of low-substituted hydroxypropyl cellulose. *H*1–*H*9 are the neurons of the hidden layer. *Y* is the output, which is the percentage of drug release in the time points of *X*1.

As Figure 1 shows, a three-layer fully connected neural network combines eight independent variables in the input layer and one response variable in the output layer. By summing the input of the previous layer and calculating the activation function, the output of the node to the next layer is calculated. The activation function used in this project is the sigmoid function described by the following equation:

(1) $$\begin{array}{c} S\left(y_{j}\right)=\;\frac{1}{1+e^{-y_{j}}}. \end{array}$$

Here, *S*(*y*_*j*_) is the output from the j-th node, and *y*_*j*_ is defined as follows:

(2) $$\begin{array}{c} y_{j}=\sum_{i=1}^{n}W_{ij}x_{i}+B_{j}, \end{array}$$

where *x*_*i*_ is the input of the *i*-th node in the previous layer. The total number of nodes is *n*, *W*_*ij*_ is the corresponding weight, and *b*_*j*_ is the bias. The artificial neural network is iteratively trained to minimize the mean square error (MSE). The gradient of the MSE performance function is used to adjust the network weights and biases until the MSE reaches 10^−5^. This study uses MATLAB R2020b version (MathWorks Inc., Natick, MA, USA) to develop and train ANN. The program automatically generates the initial weights and deviations of the network.

### 2.5. Insufficient Data Lead to Prediction Errors

Some external factors, such as the position of the tablet in the dissolution cup (the tablets always not drop in the middle of the cup are then put in), the tablet weight (the allowable tablet weight error is ±10%), the hardness of the tablet (the hardness of the same thickness is always more significant when the tablet with higher weight), and the test results of tablets with the same prescription, are always different. Therefore, there will be an error between our test value and the expected value. When the input data are the test value, the experimental error will lead to the deviation of the actual prediction. The more significant the amount of input data, the smaller the prediction error caused by experimental error. It is why the model's prediction accuracy is unstable when the data are insufficient. Therefore, most ANN applications to predict formulations will use large amounts of data to train the model and make predictions. For example, in Saman Sarraf's study, he used an ANN model to predict the betamethasone release rate, and it prepared over 80 samples. However, the input layer neurons are only 5. The prediction effect can be academically proved, but 80 experiments are enough to complete a complete orthogonal experiment in practical applications. According to the orthogonal experiment design of 5 factors and five levels, 25 experiments can result. Therefore, using a large amount of data to train the model has no practical application significance. In this project, the model should be helpful to assist formulation research and development from the beginning of the formulation project. Therefore, 21 samples with 7 influence factors were prepared. Some external factors, such as the position of the tablet in the dissolution cup (the tablets always not drop in the middle of the cup are then put in), the tablet weight (the allowable tablet weight error is ±10%), the hardness of the tablet (the hardness of the same thickness is always more significant when the tablet with higher weight), and the test results of tablets with the same prescription, are always different. Therefore, there will be an error between our test value and the expected value. When the input data are the test value, the experimental error will lead to the deviation of the actual prediction. The more significant the amount of input data, the smaller the prediction error caused by experimental error. It is why the model's prediction accuracy is unstable when the data are insufficient. Therefore, most ANN applications to predict formulations will use large amounts of data to train the model and make predictions. For example, in Saman Sarraf's study, he used an ANN model to predict the betamethasone release rate, and it prepared over 80 samples. However, the input layer neurons are only 5. The prediction effect can be academically proved, but 80 experiments are enough to complete a complete orthogonal experiment in practical applications. According to the orthogonal experiment design of 5 factors and five levels, 25 experiments can result. Therefore, using a large amount of data to train the model has no practical application significance. In this project, the model should be helpful to assist formulation research and development from the beginning of the formulation project. Therefore, 21 samples with 7 influence factors were prepared.

### 2.6. Two Methods to Solve the Problem of Unstable Prediction Result

#### 2.6.1. Effective Data Regression Method (EDRM)

Since the model is trained through multiple sets of logical data, the predicted data are mainly distributed near the actual value as long as the model is valid. First, the probability and statistics method obtains multiple prediction results of the same input dataset through multiple training and prediction. Then, the prediction result obtained after each training is used as a decision tree. If it meets the requirements, it will be retained, and if it does not meet the requirements, it will be deleted. According to statistical methods, the model calculates the standard deviation of all predicted data and then calculates the average of all predicted data. If the absolute value of the difference between the predicted value and the average value is greater than the standard deviation, the data will be automatically deleted. In this way, the model can eliminate the abnormal data generated when the predicted data converge to the optimal local solution. However, finally, we calculate the average of all the data to get an average curve. The stability of the prediction value is always decided by the number of training and prediction time.  Figure 2 shows the flowchart of EDRM in the program.

#### 2.6.2. Reference Line Regression Method (RLRM)

The second method is based on the first method and changes the screening method for abnormal data generated when the predicted data converge to the optimal local solution. First, one or multiple sets of experimental data from the training are set as reference data. In this test, depending on the number of experimental data, only one set of data was selected for testing. The reference data should also be tested by the program data screen system (see the data screen model). After each model training, the model makes predictions on this dataset, compares the prediction results with the data, and calculates the *F*2 value. When *F*2 is less than the set value (the initial *F*2 set value of this model is 65, and this value can be customized according to the project), the model is considered to converge to the optimal local solution. The program automatically recognizes it as an abnormal model and deletes it. When the number of models that meets the requirements reaches the set value (the set value is custom, and the initial set value of this model is 50), the filtered data are averaged to get the regression line. Same as EDRM, when the number of training predictions increases, the value of the curve tends to stabilize. The progress and the prediction result of formulation 3 of RLRM in the program are shown in Figure 3.

## 3. Results and Discussion

### 3.1. Results of Formulation Experiment

The percentage of ingredients in every formulation of the experiments is shown in Table 3. The experimental method is described in the chapter of materials and methods.

The dissolution test result of these formulations with the condition of 37°C in water is shown in Figure 4.

### 3.2. Prediction Result of EDRM versus RLRM

First, the first 20 sets of data are selected in the 21 sets of data to train the model. Then, the predicted value of the 21st set of data is obtained. The model is trained for 50 times and compared to the predicted values. The test results are as follows.

In Figure 5, the *x* axis is the dissolution time, and the *y* axis is the dissolution corresponding to the dissolution time.

After 50 predictions of formulation 21, it is found that the results of each test greatly vary. According to theoretical analysis, the following are the two reasons:

1. After the neural network model was trained, the model did not fully converge due to insufficient training data. In this case, the predicted value obtained by the model will be larger or smaller than the actual value. However, it is still within the usual error range.
2. Sometimes, the model prediction data will converge to a locally optimal solution. In this case, the model's predicted value will be very different from the actual value, resulting in abnormal data.

To solve these two problems, this project combines statistics and random forest methods to propose two methods.

#### 3.2.1. EDRM

The progress and the prediction result of formulation 3 of EDRM in the program are shown in Figure 6.

As shown in Figure 6, the blue line is the actual value obtained from the experiment, and the red line is the predicted value. We bring the two into the *F*2 calculation formula, and the *F*2 is 54.48, indicating that the two curves are similar. We explain that this method can solve the problem.

#### 3.2.2. RLRM

After changing the RLRM instead of EDRM for the last test, the model gives the following results.

As shown in Figure 7, the blue line is the actual value obtained from the experiment, and the red line is the predicted value. We bring the two into the *F*2 calculation formula, and the *F*2 is 62.94, indicating that the RLRM gives a better result than EDRM.

In RLRM, the choice of the reference line is significant. When the reference line is changed, the predicted value will also change. Therefore, choosing a suitable reference line will improve the prediction accuracy. The accuracy of the model's prediction is tested on the reference line: we select formulation 13, formulation 16, and formulation 21 as reference lines to predict formulation 2. The 19 sets of data other than prediction data and reference lines are all regarded as input data. The result is shown in Table 4 and Figure 8.

Comparing the two methods, the algorithm of EDRM can meet the model requirements and is more stable. The algorithm of method 2 requires higher accuracy of reference data. When there is enough standard reference data, RLRM will give better performance than EDRM.

### 3.3. Solving the Problem of the Original Data Cannot Be Used after Changing Some Excipients in the Prescription

In the actual preparation experiment process, the types of excipients in the prescription are always fine-tuned. Existing studies that predict the results of preparation experiments through neural networks only predict a single prescription by the prescription screening of the prescription ratio. If the types of excipients in the prescription are changed during the prescription optimization process, the model needs new data and retrains. The previous experimental data were wasted. The preliminary data are still available for a method designed to meet the requirements of changing the types of excipients. First, we set the auxiliary materials in all samples as input parameters, set the amount of unadded auxiliary materials to 0, and input them into the artificial intelligence model for training at the same time as other input data. In the experiment of this project, a total of 3 prescriptions were designed. Each of them has one excipient that is different from the other two to test our method's feasibility.

The actual sample size of the second formulation composition is only three groups, but there are five variables. In mathematics, it cannot be solved. Nevertheless, according to the method of the project, this problem is perfectly solved.

In the test, formulation 15 is selected as under test data, which is the second formulation composition. In EDRM, the other 20 formulation data were set as input data, and the training time was 100. For RLRM, formulation 21 was set as the reference line. The other 19 formulation data were set as input data to train the model. EDRM is used to predict formulation 15 and give the *F*2 value. The prediction result is shown in Table 5 and Figure 9.

In Table 5, the second and third columns show the formulation 15 prediction result by using EDRM and RLRM. The fourth column shows the experimental result of formulation 15.

### 3.4. Research of the Relationship between Prediction Times and the Prediction Stability

According to the above two methods, it can be found that the number of predictions is a crucial point. The following gradient experiment is designed to explore the relationship between the number of predictions and the accuracy of the model. We selected a set of data for each of the three prescriptions for testing and the unique formulation 13, formulation 16, and formulation 21 as the target prediction data values. Then, the model is trained and predicted 2 times, 10 times, and 50 times for each set of data values. Each training is repeated 10 times, and its prediction results are analyzed to calculate RSD. The experimental results are shown in Tables 6–8 and Figures 10–12.

#### 3.4.1. Formulation 21 Predicts 10 Times

The results of 10 times are given in Table 7.

#### 3.4.2. Formulation 21 Predicts 50 Times

The results of 50 times are given in Table 8.

In summary, when the number of predictions is 2, 10, and 50, the RSD values of the 10 test data are 16.37, 5.69, and 3.03. In addition, the RSD of *F*2 is 5.19, 2.50, and 1.58. When the number of predictions is only two, there was also a case where *F*2 was only 47.96. It shows that at least one data of this test converge on the optimal local solution. The test result shows that more prediction times can reduce the influence of abnormal data and the prediction error of the result.

### 3.5. Input Data Screen

In actual project applications, data with large deviations are often generated due to improper or incorrect operation of the formulation or analyst during the experiment. At this time, it is essential to filter the data. In this model, an initial was set as a training number. After input, the program will predict the input data after the initial input data, compare it with the actual input data, and calculate the *F*2 value. At this point, the *F*2 value can be calculated according to the project setting an appropriate *F*2 interval as the allowable error range. When *F*2 is not in this interval, the program will pop up a prompt. Researchers can manually delete the data. In addition, when the amount of data is large, manual screening may take more time. At this time, it can be changed to filter based on the *F*2 value automatically. The program will no longer ask whether to keep the suspected error data and delete it automatically.

## 4. Conclusions

In conclusion, it is a data prediction model that can meet the early stage of the preparation experiment and when there is only a small amount of data. When the later data are abundant, the influence of time noise becomes smaller due to the correction of a large amount of data. The prediction accuracy of the model will become higher and higher. In addition, when changing the prescription, the previous similar prescription can still be used as training data to train the new prescription model. This method also solves the problem that the preliminary research cannot be used as a basis after fine-tuning the composition of the prescription excipients. In addition, the designed model also has the input data-screening function, which immediately affects the input of abnormal data with a small amount of data and provides a basis for future high-throughput data training.

During the test, the uncontrollable noise of the experiment will affect the prediction data. The cause of the error may be the poor loading of tablets, but the prediction accuracy remains at *F*2 > 50. Compared with method 2, the algorithm of method 1 is more stable and runs faster. The prediction accuracy of RLRM is affected by the reference line. Therefore, it is better to select an optimal curve first and then use it as a reference line when using RLRM. It will improve forecast accuracy.

## Figures and Tables

**Figure 1:** The model structured by an ANN with a BP network.

**Figure 2:** The flowchart of EDRM in the program.

**Figure 3:** The flowchart of RLRM in the program.

**Figure 4:** The dissolution test result of formulations with the condition of 37°C in water.

**Figure 5:** The result of the model trained and prediction value.

**Figure 6:** The prediction result of formulation 3 of EDRM.

**Figure 7:** The prediction result of RLRM.

**Figure 8:** The contrast curve of the results.

**Figure 9:** The contrast curve of formulation 15; in summary, from the prediction results, it can be found that the value of *F*2 is over 50. It means that the similarity between the predicted curve and the actual experimental value is more significant than 90%. It shows that our method effectively solves the problem that data cannot continue training after fine-tuning the types of prescription excipients.

**Figure 10:** The comparison diagram of 10 prediction data of formulation 21 when the training time is 2.

**Figure 11:** The comparison diagram of 10 prediction data of formulation 21 when the training time is 10.

**Figure 12:** The comparison diagram of 10 prediction data of formulation 21 when the training time is 50.

**Table 1:** The comparison of related projects.

Projects	ANN model	Regression method	Input and output	Amounts of parameters and samples
This project	ANN with backpropagation network	EDRM and RLRM	Input: the factors of tablets and the time points of dissolution. Output: dissolution results in every time points.	21 samples and 7 parameters. 3 kinds of formulation composition
Yixin Chen's project [17]	No algorithm is shown in the study	The average value of 10 times prediction	Input: the factors of tablets. Output: dissolution result of a single time point	22 samples and 4 parameters
Jothi G. Kesavan's project [18]		PROC REG	Input: hardness, friability, and thickness. Output: disintegration time	23 samples and 3 parameters
Uttam MANDAL's project [19]	ANN using multilayer perceptrons	Higuchi equation	Input: the composition of tablets. Output: dissolution result of a single time point.	13 samples and 3 parameters

**Table 2:** Composition of 500 mg tinidazole tablet [15].

Ingredients	Amount
Tinidazole (TNZ)	500 mg
Microcrystalline cellulose PH 101 (PH101)	5.0%–20.0% w/w
Starch	1%–20% w/w
Croscarmellose sodium (CCNA)	0.5%–7% w/w
Hydroxypropyl methyl cellulose (HPMC)	0.5%–2% w/w
Magnesium stearate (MS)	0.5%–1.0% w/w
Low-substituted hydroxypropyl cellulose (L-HPC)	2.5%–5% w/w

**Table 3:** The first column is the number of formulation composition. The second to the eighth column consists of these seven ingredients' percentages.

Sample number	Tinidazole%	PH101%	Starch%	CCNA%	HPMC%	MS%	L-HPC%
1	76.92	9.54	9.54	3.00	0.71	1.00	0.00
2	76.92	13.39	6.69	1.00	1.00	1.00	0.00
3	76.92	10.04	10.04	1.00	1.00	1.00	0.00
4	76.92	6.86	13.72	0.50	1.00	1.00	0.00
5	76.92	6.96	13.92	0.50	0.80	1.00	0.00
6	69.44	14.03	14.03	0.50	1.70	1.00	0.00
7	69.44	9.12	18.24	0.50	1.70	1.00	0.00
8	71.43	19.64	4.91	3.00	0.55	1.00	0.00
9	71.43	19.10	4.77	3.00	0.70	1.00	0.00
10	71.43	19.89	3.98	3.00	0.70	1.00	0.00
11	71.43	19.10	4.77	3.00	0.77	1.00	0.00
12	71.43	18.30	4.57	4.00	0.77	1.00	0.00
13	71.43	19.83	3.97	3.00	0.77	1.00	0.00
14	88.62	5.32	2.66	0.00	0.53	0.30	2.66
15	88.62	3.70	1.85	0.00	0.53	0.30	5.00
16	88.62	6.31	1.58	0.00	0.53	0.30	2.66
17	71.5	17.4	5.1	5	0	1	0
18	71.5	16.5	5	6	0	1	0
19	71.5	16.4	5.1	6	0	1	0
20	71.5	15.4	5.1	7	0	1	0
21	71.5	17.4	5.1	5	0	1	0

**Table 4:** The prediction result of formulation 3 by using formulations 13, 16, and 21 as reference lines.

Time	Formulation 13	Formulation 16	Formulation 21	Experimental data
*F*2	49.11	56.96	55.30	N/A

**Table 5:** The prediction result for the formulation 15.

Time	EDRM	RLRM	Experimental data
*F*2	56.33	50.37	N/A

**Table 6:** 10 prediction results of formulation 21 when the training time set in twice.

	1	2	3	4	5	6	7	8	9	10	RSD
*F*2	58.75	56.10	63.98	60.17	60.76	63.63	47.96	64.46	65.62	60.70	5.19
Sum of RSD				16.37							

**Table 7:** 10 prediction results of formulation 21 when the training time set in 10 times.

	1	2	3	4	5	6	7	8	9	10	RSD
*F*2	62.27	63.07	68.16	67.41	61.78	64.15	64.17	60.58	65.05	61.54	2.50
Sum of RSD				5.69							

**Table 8:** 10 prediction result of formulation 21 when the training time set in 50 times.

	1	2	3	4	5	6	7	8	9	10	RSD
*F*2	66.99	62.99	64.85	63.81	66.48	66.18	66.36	64.71	65.17	62.27	1.58
Sum of RSD				3.03							

## Data Availability

The data in this work are stored by the corresponding author and are available from the corresponding author if necessary.
